The article "External Application of Traditional Chinese Medicine in the Prevention and Treatment of Nausea and Vomiting Caused by Chemotherapy of Non-Small-Cell Lung Cancer: A RCT Study" was retracted in 2023. Reasons: signs of a paper mill; compromised peer review; unreliable results or conclusions.

# External Application of Traditional Chinese Medicine in the Prevention and Treatment of Nausea and Vomiting Caused by Chemotherapy of Non-Small-Cell Lung Cancer: A RCT Study

**DOI:** 10.1155/2022/6992673

**Published:** 2022-08-04

**Authors:** Song-Jing Zhou, Lin Tang, Yong-Jun Fu, Chang-Qing Yang, Jia Shi

**Affiliations:** Department of Traditional Chinese Medicine, Hainan Provincial People's Hospital, Haikou 570311, China

## Abstract

**Objective:**

To investigate the external application of traditional Chinese medicine in the prevention and treatment of nausea and vomiting caused by chemotherapy of non-small-cell lung cancer.

**Methods:**

This is a prospective trial. A total of 114 patients with non-small-cell lung cancer who were hospitalized in our hospital from October 2020 to March 2022 were selected and randomly divided into the research group and the control group at the ratio of 1 : 1. The control group received chemotherapy + tropisetron 4 mg intravenous drip 30 minutes before chemotherapy./day × 3 days. The research group received chemotherapy + intravenous infusion of tropisetron 4 mg 30 minutes before chemotherapy, once a day for 3 days + external application of traditional Chinese medicine for 5 days. The therapeutic effects of the two groups of patients were compared.

**Results:**

After treatment, the serum creatinine, urea nitrogen, and endogenous creatinine in the research group were better than those in the control group (*t* = 15.943, 12.005, and 13.325; *P*=0.001, 0.005, and 0.005). After treatment, ALT and TBIL in the research group were superior to those in the control group (*t* = 11.583, 10.012, and 9.426; *P*=0.001, 0.002, and 0.001). After treatment, the physiological status, social/family status, emotional status, and family status of the research group were significantly better than those in the control group (*t* = 16.274, 5.379, 5.142, and 8.153; *P*=0.005, 0.000, 0.002, and 0.001). After treatment, the ECOG score and KPS score (82.46 ± 4.61) of the research group were significantly different from those of the control group (*t* = 11.913 and 9.357; *P*=0.035 and 0.001). The effective rate (*χ*^2^ = 11.724; *P*=0.000) of the research group was higher but the incidence of adverse reaction (*χ*^2^ = 4.294; *P*=0.001) was lower than that of the control group.

**Conclusion:**

External application of traditional Chinese medicine can significantly reduce nausea and vomiting caused by chemotherapy of non-small-cell lung cancer and can improve the patient's body and quality of life, which is worthy of clinical research and promotion.

## 1. Introduction

In recent years, the mortality and disability rate of malignant tumors has remained high, which seriously threatens human health. Lung cancer including non-small-cell lung cancer (NSCLC) is the second most common cancer and the leading cause of cancer death in the USA. Approximately 247,270 new cases of lung cancer are estimated to occur in 2020, with 130,340 male cases and 116,930 female cases. The greatest risk factor for development of lung cancer is tobacco use. Secondhand smoking has also been shown to increase the risk of lung cancer by as much as 26% [1]. Other risk factors for lung cancer include asbestos exposure, family history of lung cancer, and exposure to toxic substances, including polycyclic aromatic hydrocarbons, heavy metals, and radon gas. According to the latest statistics, the death of malignant tumors accounts for 23.91% of all deaths among residents. At present, chemotherapeutic drugs can effectively control the growth of tumor cells. Chemotherapy is still an effective means of modern medicine for the treatment of malignant tumors. However, while killing tumor cells, chemotherapeutic drugs often cause different degrees of nausea and vomiting and other gastrointestinal toxic reactions. Patients are unable to eat, and some even give up chemotherapy for fear of gastrointestinal reactions [1–3]. This study externally applied self-made chemotherapy antiemetic patches, such as Zhongwan, Neiguan, Zusanli, Yongquan, and other acupoints to prevent and treat nausea and vomiting. This operation is easy for patients to accept and clinical implementation with simple and convenient operation profile. This article discusses the value of external application of traditional Chinese medicine in the prevention and treatment of nausea and vomiting caused by chemotherapy of non-small-cell lung cancer.

## 2. Materials and Methods

### 2.1. Participants

This is a prospective trial. A total of 114 patients with non-small-cell lung cancer who were hospitalized in our hospital from October 2020 to March 2022 were enrolled as per the inclusion criteria. The eligible participants were randomly divided into the research group and the control group with 57 cases in each group at the ratio of 1 : 1. All patients in this study gave informed consent, and the patients themselves or their family members signed the relevant consent forms. The baseline data of the included subjects are detailed in Table 1. This study has been reviewed and approved by the Medical Ethics Committee of the Hainan Provincial People's Hospital (no. #1733119, clinical study registration number: ChiCTR2300061257).

#### 2.1.1. Inclusion Criteria

Inclusion criteria were as follows: ① age from 18 to 80 years; ② patients with malignant tumors diagnosed by pathology and those with gastrointestinal reactions such as vomiting and nausea after one-stage chemotherapy; ③ patients without contraindications to chemotherapy and with KPS score greater than 70 points; ④ blood routine and liver and kidney function are basically normal; ⑤ those who are informed and willing to receive treatment.

#### 2.1.2. Exclusion Criteria

Exclusion criteria were as follows: ① patients with mental illness; ② vomiting caused by other reasons other than chemotherapy; ③ pregnant or breastfeeding women; ④ patients with severe heart, liver, and kidney dysfunction or abnormal bone marrow function.

### 2.2. Methods

#### 2.2.1. Control Group

The control group was given chemotherapy + tropisetron 4 mg intravenous infusion 30 minutes before chemotherapy 1 time/day for 3 days.

#### 2.2.2. Research Group

The research group was administered chemotherapy + intravenous infusion of tropisetron 4 mg 30 minutes before chemotherapy, once a day for 3 days + external application of traditional Chinese medicine for 5 days. The external application of traditional Chinese medicine on the acupoints of Zhongwan, Guanyuan, Zusanli (double), and Yongquan (double) was started from 2 days before the application of chemotherapy drugs to the third day of chemotherapy, once a day for 4 hours each time. Among them, the external medicine was composed of Pinellia, tangerine peel, Poria, Atractylodes, Kou Ren, cooked aconite, cinnamon, dried ginger, Evodia, and cloves in equal proportions. We form a bolus weighing about 3 g and fix the bolus on the selected acupoint with a 6 × 6 nonwoven blank sticker. The acupoints were applied externally from 1 day before the application of chemotherapy drugs to the 4th day of chemotherapy, once a day for 4 hours each time.

### 2.3. Observation Indicators

#### 2.3.1. Efficacy

(1) Main efficacy indicators were the frequency, degree, and duration of nausea and vomiting. (2) Secondary efficacy indicators were nausea and vomiting interval, chemotherapy drug dose reduction, the proportion of interruption or withdrawal, and quality of life score.

#### 2.3.2. Safety

(1) Records of adverse reactions included the following: constipation, dizziness, headache, abdominal distension, and diarrhea. (2) Blood routine, urine routine, stool routine, liver and kidney function, and electrocardiogram.

#### 2.3.3. Antiemetic Efficacy

Complete control (CR) (no vomiting), partial control (PR) (vomiting 1 to 2 times/d), mild control (MR) (vomiting 3 to 5 times/d), and no control (F) (vomiting > 5 times/d) were observed. The total effective control rate was CR + PR. Complete remission rate refers to the ratio of cases with normal eating and no nausea and vomiting to the total number of cases. Effective rate refers to the proportion of cases with no nausea and mild nausea, no effect on eating, complete relief of vomiting, and partial relief to the total number of patients.

Nausea and vomiting index evaluation: according to the anticancer drug toxicity standard prepared by the World Health Organization, ① 0 degree denotes no nausea and vomiting; ② I degree denotes nausea and no vomiting; ③ II degree denotes nausea with mild vomiting; ④ III degree denotes severe vomiting; and ⑤ M degree denotes vomiting is difficult to control. Nausea profile (NP) assessment: NP is divided into 3 parts of symptoms: ① physical discomfort: dizziness, weakness, fatigue, sweating, and other accompanying symptoms; ② gastrointestinal reactions: evaluation of the manifestation and degree of nausea, vomiting, and stomach discomfort; and ③ emotional discomfort: assessment of nervousness, anxiety, disappointment, fear, and other negative emotions. The higher the score, the more severe the above symptoms.

The American Cancer Quality of Life Scale (FACT-L4.0) was used to evaluate the impact of treatment regimens on the quality of life of patients.

Scoring and evaluation were performed according to the Eastern Cooperative Oncology Group Physical Condition Scale (ECOG) and KPS. By comparing the changes of ECOG/KPS values before and after treatment, the influence of the treatment plan on the patient's physical state was evaluated.

### 2.4. Statistical Analysis

The data analysis was done with SPSS21.0 software package; the count was tested by the *χ*^2^ test and expressed as %, and the measurement was tested by the *t*-test and expressed as $\bar{x}\pm s$. *P* < 0.05 indicated that the difference is of statistical significance.

## 3. Results

### 3.1. Comparison of Renal Function between the Two Groups before and after Treatment

There was no significant difference in renal function between the two groups before treatment. After treatment, the serum creatinine in the study group was 564.14 ± 93.22 and in the control group was 235.84 ± 65.15; the urea nitrogen level in the study group was 24.33 ± 8.14 and in the control group was 15.12 ± 8.41; the endogenous creatinine level in the study group was 15.34 ± 8.22 and in the control group was 23.41 ± 10.82; the differences were significant (*t* = 15.943, 12.005, and 13.325; *P*=0.001, 0.005, and 0.005) (Table 2).

### 3.2. Comparison of Liver Function between the Two Groups before and after Treatment

Before treatment, there was no significant difference in the liver function between the two groups. After treatment, ALT level was 30.92 ± 11.18, AST level was 34.17 ± 9.19, and TBIL level was 21.28 ± 6.16 in the study group. In the control group, ALT level was 38.58 ± 12.16, AST level was 41.19 ± 8.43, and TBIL level was 26.05 ± 9.83, and the differences were significant (*t* = 11.583, 10.012, and 9.426; *P*=0.001, 0.002, and 0.001) (Table 3).

### 3.3. Comparison of Quality of Life before and after Treatment between the Two Groups

Before treatment, the physiological status (25.50 ± 3.50), social/family status (28.40 ± 1.10), emotional status (27.26 ± 2.20), and family status (30.40 ± 1.10) of the research group were comparable to the control group's physiological status (26.61 ± 2.11), social/family status (28.51 ± 2.2), emotional status (27.43 ± 1.21), and family status (30.41 ± 0.11), and the differences were insignificant (*t* = 7.943, 9.536, and 6.451; *P*=0.564, 0.826, 0.624, and 0.150). After treatment, the physiological status (16.40 ± 1.20), social/family status (17.60 ± 0.40), emotional status (18.94 ± 1.60), and family status (20.50 ± 1.10) of the research group were better than the control group's physiological status (20.21 ± 6.41), social/family status (20.11 ± 1.51), emotional status (20.85 ± 1.31), and family status (22.81 ± 1.21), and the differences were significant (*t* = 16.274, 5.379, 5.142, and 8.153; *P*=0.005, 0.000, 0.002, and 0.001) (see Table 4 for details).

### 3.4. Comparison of Physical Condition Scores between the Two Groups before and after Treatment

Before treatment, the ECOG score (3.59 ± 0.12) and KPS score (60.25 ± 4.32) in the research group were comparable to the ECOG score (3.13 ± 0.14) and KPS score (60.72 ± 4.38) in the control group (*t* = 9.548 and 8.736, *P*=0.682 and 0.748). After treatment, the ECOG score (1.47 ± 0.52) and KPS score (82.46 ± 4.61) of the research group were significantly different from the ECOG score (2.16 ± 0.89) and KPS score (78.24 ± 4.56) of the control group (*t* = 11.913 and 9.357; *P*=0.035 and 0.001) (Table 5).

### 3.5. Comparison of Antiemetic Efficacy between the Two Groups of Patients

The effective rate of the research group was significantly better than that of the control group (73.68% (42/57) vs 52.63% (30/57)), with a significant difference (*χ*^2^ = 11.724, *P*=0.000). The total effective rate of the research group was significantly better than that of the control group (91.23% (52/57) vs 80.70% (46/57)), with a significant difference (*χ*^2^ = 9.458, *P*=0.015) (Table 6).

### 3.6. Comparison of the Incidence of Adverse Reactions between the Two Groups of Patients after Treatment

The incidence of adverse reactions in the research group was lower than that in the control group (31.58% (18/57) vs 47.37% (27/57)), with a significant difference (*X*^2^ = 4.294, *P*=0.001) (Table 7).

## 4. Discussion

Lung cancer remains the leading cause of cancer-related death in many countries, as many patients are diagnosed at an advanced stage (III or IV). Surgery alone leads to poor overall survival in hospitalized patients with stage III NSCLC, most of whom have tiny distant metastases. Due to the dismal 5-year survival rate of patients with stage IIIA-N2 NSCLC who underwent surgical resection alone, treatment of advanced NSCLC should control local and microscopic systemic disease [4, 5]. One way to improve surgical outcomes is to give chemotherapy before or after surgery. Over the past two decades, many clinical studies have focused on developing optimal adjuvant or neoadjuvant chemotherapy regimens and/or radiotherapy for advanced lung cancer that can be combined with surgery. Treatment options for NSCLC are largely based on the stage of the cancer. However, other factors, such as a person's health, lung function, and cancer characteristics, are also taken into account. The therapeutic goals of NSCLC are to prolong survival and control disease-related symptoms [6–8]. For patients who are not candidates for molecularly targeted therapy, similar survival outcomes can be achieved with various platinum doublets and these are recommended by current National Comprehensive Cancer Network (NCCN) guidelines. In addition, the most commonly used chemotherapeutic agents have different toxicity profiles and thus toxicity profiles are involved in determining treatment selection, patient tolerance to chemotherapy, and treatment success rates [9]. Although most cancer patients prefer to take an active or shared role in decision-making, no clear clinical guidelines have been published on how to obtain and integrate their preferences for side effects in treatment decisions.

In cancer patients, chemotherapy-induced nausea and vomiting (CINV) is a common adverse effect that affects not only quality of life but also treatment outcomes. The main cause of nausea and vomiting during chemotherapy is that chemotherapy drugs stimulate the gastrointestinal mucosa. When chemotherapy drugs accumulate in the intestinal cavity of patients, they stimulate enterochromaffin cells to release neurotransmitters such as serotonin, which combine with serotonin at the vagus nerve terminals in the abdominal cavity. Subsequently, it generates nerve impulses and stimulates the emesis center on the dorsolateral side of the reticular structure of the medulla oblongata in the brainstem, causing vomiting. It is important to address these issues from both preventive and therapeutic perspectives so that patients can adhere to their treatment regimen. Nausea and vomiting are divided into 5 different types, and the main drug options for prevention and treatment include 5-HT3 receptor antagonists, NK1 receptor antagonists, and corticosteroids. Other drugs used (but to a lesser extent) include dopamine antagonists, benzodiazepines, cannabinoids, and olanzapine [10, 11]. In addition, those patients who express interest in alternative or nondrug therapies may also have options. Risk factors for developing nausea and vomiting can be classified as patient-related or treatment-related factors.

Nausea and vomiting are the most common side effects of chemotherapy drugs, which may lead to dehydration, electrolyte disturbances, and malnutrition, and negatively affect patients' treatment compliance. 70% to 80% of cancer patients will develop CINV without appropriate antiemetic intervention. Therefore, effective management of chemotherapy-induced nausea and vomiting (CINV) is beneficial to patient compliance and quality of life [12]. For CINV, antiemetics divided into the following classes are recommended as follows: 5-HT3 serotonin receptor antagonists, tachykinin NK1 receptor antagonists, steroids, olanzapine, dopamine receptor antagonists, and benzodiazepines class of drugs. However, full control of CINV remains unresolved. In addition, the expensive cost and side effects of antiemetics, including constipation, headache, and hiccups, also indicate that CINV still needs better treatments [13]. Acupuncture, acupressure, massage, and moxibustion are all safe medical procedures with minimal side effects for CINV. The National Institutes of Health (NIH) consensus statement recommends acupoint stimulation as a complementary intervention for CINV prevention. The Society for Oncology Nursing also considers acupoint stimulation as a promising intervention for the treatment of CINV [14]. A previous systematic review showed that acupoint stimulation reduces the incidence of acute vomiting. In this study, the effective rate of the research group was 73.68% (42/57), which was significantly better than that of the control group, 52.63% (30/57). The total effective rate of the study group was 91.23% (52/57), which was significantly better than that of the control group, 80.70% (46/57). Data show that external application of traditional Chinese medicine on acupoints can reduce the incidence of nausea and vomiting in patients undergoing chemotherapy. Physiologically, the spleen and stomach are the foundation of essence. However, chemotherapy drugs are classified as “drug poisons” and “drug evils,” which lead to the disharmony of the stomach and the upward reversal of stomach qi, resulting in a series of gastrointestinal reactions such as nausea, vomiting, and loss of appetite in patients after chemotherapy [8]. “Medical Origins” mentions “the external TCM application blocks its qi, enables the medicinal properties enter its internal organs from the pores, pass through the meridians, between the skin, muscles, and bones, via pasting it with ointment.” The external application of traditional Chinese medicine uses meridians and acupoints as carriers and channels, so that the medicine directly acts on the relevant organs, and stimulates the effect of the medicine through the sensitivity and amplification effect of the meridians and acupoints on the medicine.

The limitations of this study need to be addressed. First, this pilot study might not have sufficient total sample size to obtain reliable results. Future studies should endeavor to recruit larger sample sizes to further verify the treatment effects.

To sum up, external application of traditional Chinese medicine can significantly reduce nausea and vomiting caused by chemotherapy of non-small-cell lung cancer and can improve the body and quality of life of patients, which is worthy of clinical research and promotion.

## Figures and Tables

**Table 1:** Basic profiles of patients.

General	Research group	Control group	*t* value/*χ*^2^ value	*P* value
Number of cases	57	57		

Age	59.38 ± 1.29	60.15 ± 2.03	1.812	0.074

Sex			0.202	0.653
Male	28	27		
Female	29	30		

Nation			2.124	0.000
Han nationality	54	55		
Others	3	2		

Smoking history			0.521	0.000
None	10	7		
Less than 10 years	25	24		
10+ years	22	26		

Drinking history			0.142	0.003
None	21	23		
Less than 10 years	24	24		
10+ years	12	10		

**Table 2:** Comparison of renal function in the two groups before and after treatment ($\bar{x}\pm s$).

Group	Case	Serum creatinine (*μ*mol/L)		Urea nitrogen (mmol/L)		Endogenous creatinine (ml/min)	
		Before treatment	After treatment	Before treatment	After treatment	Before treatment	After treatment
Control group	57	945.63 ± 129.81	564.14 ± 93.22	47.13 ± 11.52	24.33 ± 8.14	10.51 ± 6.93	15.34 ± 8.22
Research group	57	953.81 ± 133.63	235.84 ± 65.15	48.64 ± 10.42	15.12 ± 8.41	11.12 ± 5.83	23.41 ± 10.82
*t*		2.019	15.943	1.631	12.055	1.461	13.325
*P*		0.245	0.001	0.031	0.005	0.102	0.005

**Table 3:** Comparison of the liver function between the two groups before and after treatment ($\bar{x}\pm s$).

Group	Case	ALT (U/L)		AST (U/L)		TBIL (*μ*mol/L)	
		Before treatment	After treatment	Before treatment	After treatment	Before treatment	After treatment
Control group	57	95.31 ± 32.06	38.58 ± 12.16	72.38 ± 11.43	41.19 ± 8.43	38.18 ± 11.93	26.05 ± 9.83
Research group	57	93.74 ± 37.91	30.92 ± 11.18	75.12 ± 12.16	34.17 ± 9.19	37.26 ± 12.17	21.28 ± 6.16
*t*		2.354	11.853	1.557	10.012	1.570	9.426

**Table 4:** Comparison of quality of life before and after treatment in the two groups ($\bar{x}\pm s$).

Group	Physiological condition		Social/family status		Emotional status		Family status	
	Before treatment	After treatment	Before treatment	After treatment	Before treatment	After treatment	Before treatment	After treatment
Research group	25.50 ± 3.50	16.40 ± 1.20	28.40 ± 1.10	17.60 ± 0.40	27.26 ± 2.20	18.94 ± 1.60	30.40 ± 1.10	20.50 ± 1.10
Control group	26.61 ± 2.11	20.21 ± 6.41	28.51 ± 2.2	20.11 ± 1.51	27.43 ± 1.21	20.85 ± 1.31	30.41 ± 0.11	22.81 ± 1.21
*T*	7.943	16.274	9.538	5.379	6.451	5.142	10.221	8.153
*p*	0.564	0.005	0.826	0.000	0.624	0.002	0.150	0.001

**Table 5:** Comparison of physical conditions before and after treatment in the two groups (points, $\bar{x}\pm s$).

Group	ECOG score		KPS score	
	Before treatment	After treatment	Before treatment	After treatment
Research group (*n* = 57)	3.59 ± 0.12	1.47 ± 0.52	60.25 ± 4.32	82.46 ± 4.61
Control group (*n* = 57)	3.13 ± 0.14	2.16 ± 0.89	60.72 ± 4.38	78.24 ± 4.56
*T*	9.548	11.913	8.736	9.357
*P*	0.682	0.035	0.748	0.001

**Table 6:** Comparison of antiemetic efficacy between the two groups of patients (cases, %).

Group	Complete control (CR)	Partial control (PR)	Slight control (SR)	No control (F)	Obvious efficiency	Total effective control rate
Research group (*n* = 57)	20 (35.09)	22 (38.60)	10 (17.54)	5 (8.77)	42 (73.68)	52 (91.23)
Control group (*n* = 57)	12 (21.05)	18 (31.58)	16 (28.07)	11 (19.30)	30 (52.63)	46 (80.70)
*χ* ^*2*^		—			11.724	9.458
*P*		—			0.000	0.015

**Table 7:** Comparison of adverse reactions (cases).

Group	Case	Constipation	Dizziness/headache	Bloating/diarrhea	Incidence (%)
Research group	57	8	10	9	47.37
Control group	57	5	8	5	31.58
*X* ^*2*^	—		4.294		
P	—		0.001		

## Data Availability

All data generated or analysed during this study are included within this article.
